# Analysis of the influence of enterprise managers’ overconfidence on the overinvestment behavior of listed companies under the media reports

**DOI:** 10.3389/fpsyg.2022.1018189

**Published:** 2022-10-18

**Authors:** Michael So

**Affiliations:** Faculty of Business and Management, BNU-HKBU United International College, Zhuhai, China

**Keywords:** external governance, marketization process, media reports, enterprise overinvestment, managers’ overconfidence

## Abstract

At present, there is a common overinvestment behavior among listed companies in various countries, which seriously reduces the overall resource allocation efficiency of the market. With the rise of behavioral finance, it has become a new direction to study the influence of managers’ “irrational characteristics” on enterprise overinvestment. With the rapid rise of the media industry, media reporting, as an external governance mechanism, supplements the capital market supervision system and has a huge impact on the investment behavior of enterprises. How media reports affects overinvestment and whether it can curb overinvestment caused by managers’ overconfidence is still worthy of further study. This paper took 6,012 A-share listed companies from 2013 to 2021 as samples, and based on the perspective of “media reports,” studies the impact of managers’ overconfidence on overinvestment; explores whether positive and negative media reports have a moderating effect between overconfidence and overinvestment; studies the moderating effect of media reports under different marketization processes. Empirical conclusions: (1) Managers’ overconfidence will lead to overinvestment of enterprises. (2) Positive media reports will aggravate the overinvestment caused by managers’ overconfidence; negative reports can inhibit the overinvestment caused by managers’ overconfidence. (3) In regions with higher marketization, positive media reports play a more significant role in aggravating overconfidence and leading to overinvestment; in regions with lower marketization, negative reports play a stronger role in restraining overconfidence and overinvestment.

## Introduction

Investment activities play an important role in enterprise management. Enterprise investment is not only related to the short-term operation of the enterprise, but also to the long-term strategy of the enterprise, as well as the performance and future sustainable development of the enterprise (Dejuanbitria and Morasanguinetti, 2021; Sharpe and Suarez, 2021). In the current listed companies, the phenomenon of overinvestment is more serious than underinvestment (Li et al., 2020). During the 9-year period from 2006 to 2014, Dongfang Electric’s net cash flow from enterprise investment activities was all less than zero. In such a financial predicament that cannot make ends meet, Dongfang Electric still conducts large-scale expansion (Mitan et al., 2021). Overinvestment has caused Dongfang Electric to repeatedly fall into financial crisis and shut down a large number of huge projects. In 2017, Wanda Hotel Development, a subsidiary of Wang Jianlin, issued an announcement to suspend all investment in Spain and sell all the shares of Spain Building (Yang et al., 2017). Wang Jianlin’s investment in Spain ended with a loss of 200 million yuan, which means that Wanda completely lost to Spain. Due to the lack of scientific evaluation of investment projects, blind expansion and excessive investment led to the failure of Wanda’s second overseas investment and acquisition in 2017.

In today’s era of big data networks, the media industry has risen rapidly. The behavior and development status of listed companies are one of the main contents of media attention and reports (Kim et al., 2021). Figure 1 counts the number of reports on Shanghai and Shenzhen A-share listed companies by eight authoritative mainstream media such as China Securities Journal during the period from 2013 to 2021. It can be seen that whether it is positive or negative, the number of media reports on companies is on the rise (Du and Li, 2021). The media has become an important bridge and link between public investors, enterprises and the capital market. The voice of the media will have a huge impact on the decision-making and development of enterprises and the investment direction of investors (Johnson et al., 2022).

**FIGURE 1:** Times of mainstream media reports on listed companies from 2013 to 2021.

China’s Yinguangxia Trap, melamine milk powder and other incidents have made society and enterprises understand the role of the media (Halawani et al., 2020; Klein et al., 2021). On February 15, 2019, China Securities Journal and other media exposed that there are major food safety problems in Sanquan dumplings. After February 15, the number of relevant media reports began to increase. As of February 18, the number of relevant media reports exceeded 3,000, and it was still on the rise. This negative news led to a rapid decline in the stock and sales of Sanquan Foods, resulting in heavy losses, and major platforms removed related products one after another. More seriously, the reputation and value of the company have been greatly affected, and it has also greatly slowed down the further investment of Sanquan Group. In just a few days, the stock price of Sanquan Foods fell by 5%. According to the financial report data released by Sanquan Foods, the operating income of dumplings in the first half of the year fell by as much as 17.59% year-on-year, which led to the large-scale removal of Sanquan products online and offline (Chen and Chen, 2022).

Traditional financial theories are based on the premise and assumption that managers are completely rational people, and often attribute overinvestment to principal-agent conflicts (Kariuki et al., 2020; Sun et al., 2021). However, in real economic activities, managers are not “completely rational,” and individual managers’ behavioral decisions and judgments often deviate from rationality, and subjective errors often occur due to psychological factors (Wong, 2020; Zhang and Chen, 2020; Gupta et al., 2021). With the deepening of research, psychology, finance and management are gradually combined, and factors related to the irrational and heterogeneous characteristics of managers have begun to be taken into account (Bortoli et al., 2019). The rise of behavioral finance has made up for the defect of traditional finance that is based on the premise of a completely rational economic man (Araújo Júnior et al., 2019; Wu et al., 2022a). Roll (1986) is the pioneer of introducing “overconfidence” in the study of business management issues, and believes that overconfidence psychology will directly affect managers’ investment decisions, and eventually lead to overinvestment. In recent years, many scholars have carried out in-depth research from the point of view of overconfidence, and the research on the relationship between overconfidence and overinvestment has gradually matured (Wan et al., 2021; Yong et al., 2021). But how exactly is the variable overconfidence measured? Does it necessarily lead managers to make overinvestment decisions? These issues still deserve further exploration.

Existing literature rarely studies the combination of managerial overconfidence, media reports, and overinvestment. Can media reports restrain and regulate excessive investment behaviors caused by irrational psychology? Do positive and negative reports have different effects on overinvestment caused by managers’ irrational psychology? There is no consistent conclusion on these issues yet, and they are still worthy of in-depth analysis and discussion. In addition, many countries have vast territory and many regions, and are in the critical stage of market economy transformation, and the marketization process varies greatly. Under different marketization processes, media reports will have different responses to enterprises and society (Akbar et al., 2022). Therefore, based on the perspective of media reports, this paper explores the relationship between managers’ overconfidence and enterprise overinvestment. In addition, this paper includes the marketization process into the research scope, and discusses the role and impact of positive and negative media reports on the overinvestment caused by managers’ overconfidence under different degrees of marketization process.

Section is “Introduction,” which points out the research background and significance. Section is “Literature review,” which analyzes the research achievements and deficiencies of domestic and foreign literature, and lays the foundation for the research design of the following. Section “Research hypothesis” carries on the theoretical analysis and puts forward the research hypotheses. This part firstly analyzes related content such as overconfidence, overinvestment, media reports and marketization process, and then puts forward three hypotheses in this paper. Section “Research design” is the design of the research. This part designs the empirical research in this paper, including data sources, selection of variables, and the design and establishment of empirical models. Section “Empirical test and result analysis.” The three hypotheses of this paper are verified by a series of statistical methods, and the robustness test is carried out. Finally, the results are analyzed and explained in detail. Sections “Discussion” and “Conclusion,” respectively. On the basis of empirical test and result analysis, this paper puts forward relevant policy suggestions from the enterprise, media and government levels to improve the efficiency of enterprise investment. Finally, the shortcomings of this paper are summarized and future prospects are proposed.

## Literature review

### Overconfidence and overinvestment

In the early literature on overinvestment, most of them were based on principal-agent theory, and did not pay attention to the impact of managers’ own irrational behavior on the investment decision and development of enterprises. Mu et al. (2020) found that overconfident managers lack the ability to rationally analyze, and often misjudge the project’s net present value and rate of return, resulting in overinvestment. In addition, considering the effect of manager gender on this relationship, the overinvestment caused by overconfidence of male managers will be more serious (Liu, 2022). Because male managers have more aggressive venture capital preferences than female managers, and analyst tracking can moderate irrational behaviors caused by overconfidence (Valaskova et al., 2021). Wan et al. (2022) focused on the relationship between overconfidence and overinvestment under different property rights. The argument shows that many of the investment expansion activities of private enterprises are caused by the overconfidence of managers, which is related to the more restrictions on investment and the greater social responsibility of state-owned enterprises.

But not all scholars agree that the impact of overconfidence on business is negative. Managers with overconfidence tend to have the spirit of unyielding, innovative and enterprising spirit, which will also bring positive effects to the enterprise to a certain extent. Hijjawi et al. (2021) believes that overconfident managers also have a positive side for companies. Overconfident managers can more accurately identify high-yield investment opportunities. Ying (2022) believes that managers’ overconfidence has a positive impact on the company’s investment level. Mirzaei and Samet (2022) also believe that overconfident managers tend to have stronger insight and more professional financial capabilities, and maximize the benefits from investment.

### Media reports and overinvestment

The media is the bridge between enterprises and the public, and influences enterprise investment decisions mainly through three channels: Information efficiency mechanism, pressure and supervision mechanism, and reputation mechanism (Al-Dmour et al., 2022). First, the media transmits enterprise information to the public in a timely manner, which can reduce the information asymmetry between the two parties and enable the public and investors to make correct investment decisions from a fair and comprehensive perspective. Second, through the exposure of the media, the society strengthens the visible supervision of various regulatory departments through this invisible supervision, which will cause certain pressure on the managers of the exposed enterprises, and also bring a warning effect to other enterprises. Third, negative media reports can put a company in a dilemma of public opinion and reputation. Under pressure from the media, management strives to improve enterprise governance, enhance the company’s reputation, and save its image in the minds of the public and investors (Burke, 2022; Ed-Dafali et al., 2022; Zhao et al., 2022b).

O’Neill and Qu (2010) and Li et al. (2018) were the first to study the relationship between media reports and enterprise governance in a theoretical and systematic manner. They selected the 50 worst boards as rated by Boards magazine in 2004 for the study sample and found that media reports draws public attention. Among them, negative reports will have a great negative impact on the reputation of managers, prompting managers to effectively reduce overinvestment behaviors and make decisions that will weaken enterprise value (Lu, 2022). In terms of reputation mechanism, Li et al. (2019) and Poursoleyman et al. (2022) pointed out that the invisible supervision of the media will prompt managers to improve the investment efficiency and governance level of enterprises. Through media reports, it is possible to urge the administrative department to intervene to conduct more effective supervision, thereby reducing the irrational investment behavior of enterprises, restraining excessive investment, and achieving the effect of enterprise governance (Lee et al., 2022).

He et al. (2020) concluded that the role of the media comes from two mechanisms: one is the reputation mechanism. If an enterprise is exposed by the media, it will seriously affect the reputation and image of enterprise managers. In order to save their own reputation and enterprise image, managers will improve their decision-making ability (Wu et al., 2022b). The second is the role of information transmission. If there is no media, a lot of information about the enterprise cannot be transmitted to the public and investors, and serious information asymmetry will lead to investors unable to accurately assess the value of the enterprise (Indremo et al., 2022). Similar to the reputation mechanism, Su and Alexiou (2020) from the perspective of earnings management focused on the mechanism by which media reports would generate market pressure on executives, thereby improving enterprise governance (Burke, 2022).

There is no consensus on the relationship between media reports and enterprise overinvestment. Cui and Shi (2017) combined emotion theory and believed that media reports and exposure would attract the attention of many investors, stimulate investor sentiment, stimulate their investment intention and investment interest, and lead to further overinvestment by enterprises. Choiriah et al. (2021) found that despite frequent media reports on relevant news, it did not alleviate the tunnel behavior of major shareholders and did not improve the company’s investment efficiency. Huang et al. (2022) started from managers’ emotions and concluded that positive media reports will aggravate managers’ overestimation of their own abilities and thus make overinvestment. However, the results of the study found that the impact of negative media reports was actually minimal. However, Greo (2021) and Mundi and Kaur (2022) believe that the media does not have a unilateral impact on investment efficiency, but has both positive and negative impacts. Media reports can attract managers’ attention, improve investment prudence, and make more rational investments. However, some negative reports or news reports with exaggerated elements will affect managers’ emotions, shake managers’ confidence, and reduce investment efficiency. Blair et al. (2022) verified the market pressure hypothesis of the media from an audit perspective. The media can enhance the power of external audit, reduce the motivation of enterprise profit management, and effectively realize the role of enterprise governance.

### Overconfidence, media reports, and overinvestment

Regarding how to alleviate and alleviate the problem of overinvestment caused by overconfidence, most scholars study whether there is a moderating effect in combination with the internal enterprise governance mechanism of the company, and there are few studies on the relationship between the three from the external perspective of media reports. At present, only Huang et al. (2022) and Zhao et al. (2022a) have conducted research on the relationship between the three and reached similar conclusions, but they are only limited to negative media reports. Zhao et al. (2022a) conducted a study on A-share listed companies from 2009 to 2018 and found that negative media reports can play a positive role, reduce managers’ overconfidence, and have a certain negative adjustment to low-efficiency investment. Huang et al. (2022) also analyzed that negative reports as a moderating variable can reduce the positive correlation between overconfidence and overinvestment, and further divide the nature of property rights. It is found that negative media reports have a stronger inhibitory effect on state-owned enterprises than non-state-owned enterprises.

## Research hypothesis

### Impact of managers’ overconfidence on enterprise overinvestment

With the rise of behavioral finance, psychological factors are applied to economic management analysis, and many economic phenomena have more reasonable explanations. Overconfidence, as a very widespread and ubiquitous irrational psychology, has been deeply valued and studied by scholars at home and abroad. Roll first pioneered the “arrogance theory,” arguing that managers will be driven by overconfidence and prefer to expand abroad, resulting in excessive investment behavior. Huang et al. (2022) expanded the scope of enterprise managers from a single manager to the entire company management, and found that the two are still positively correlated. Greo (2021) and Mundi and Kaur (2022) pointed out that managers with overconfidence will be keen on enterprise expansion strategies and realize enterprise expansion by increasing investment in mergers and acquisitions, but the result will increase the possibility of companies falling into financial crisis. Blair et al. (2022) refined the scope of investment and defined it as the investment in fixed assets by enterprises. The results found that the higher the level of managers’ overconfidence, the more investment in fixed assets by enterprises. Managers’ confident mentality has a significant effect on investment decisions, and when the highest level of self-confidence is reached, that is, overconfidence, it will lead to alienation of enterprise investment behavior and overinvestment (Kunjal et al., 2021; Akbar et al., 2022).

When the net present value of an investment project is positive, the project can be initially identified as a project that can be invested; on the contrary, the project is likely to be a negative-return project and should not be invested. As an important decision maker in the company’s investment activities, managers will have a certain sense of superiority, and their decisions will be greatly affected by their own psychological factors. managers’ overconfidence usually have high investment enthusiasm and preferences, are overly optimistic about investment prospects, overly affirm and trust their own judgments, and ignore the possibility of investment failure and market risks (Jiang and Akbar, 2018). Such a mental state will lead managers to have a stronger investment intention and make wrong judgments and decisions. On the other hand, managers driven by their own interests and their desire to build a “business empire” will further encourage their willingness to invest blindly, leading to overinvestment. At the same time, due to the existence of information asymmetry, shareholders cannot supervise the behavior of managers at all times, and the purpose behind managers’ decisions is often difficult to detect. Managers lack necessary constraints when making investment decisions, which further leads to overinvestment (Xu and Liu, 2020). Therefore, this paper proposes the hypothesis H1:

Hypothesis H1: managers’ overconfidence leads to overinvestment in the enterprises.

### Moderating effect of media reports on managers’ overconfidence and overinvestment

With its own advantages, the media has built a bridge of communication between enterprises and investors, which can effectively alleviate agency conflicts and information asymmetry to a large extent, improve the overall resource allocation efficiency of the market, and play a role in enterprise governance. Media reports will greatly affect the investment efficiency of enterprises. The media timely and objectively transmit the information of the enterprise to the public and investors. Investors will screen and judge the information and then make a decision whether to invest or not. Enterprise managers will further make investment decisions based on market reactions (Bulathsinhalage and Pathirawasam, 2017). In addition, managers determine the investment direction of enterprises, and managers’ psychology will largely influence their investment decisions (Fan et al., 2022). In this ever-changing information age, the media industry is developing rapidly, and the media can timely report the information and status of various enterprises in the capital market by virtue of their advantages such as large influence and fast information transmission speed. The media reports on enterprises will have an important impact on managers’ psychology, especially overconfidence, which in turn affects enterprise managers’ investment decisions and enterprise investment efficiency, becoming one of the external governance mechanisms of enterprises (Cragun et al., 2019; Ahmed et al., 2020; Gao et al., 2021).

The effect mechanism of media reports on managers’ overconfidence and overinvestment is mainly through the media’s supervision mechanism and reputation mechanism. According to the emotional color of media reports, there are two types of media reports: positive reports and negative reports. Different media reports have different influences on managers’ psychology, which will cause enterprise managers to make different investment decisions (Brown et al., 2009). Therefore, this paper studies the impact on enterprise overinvestment from two types of media reports.

The media’s positive reports on the enterprise are often a kind of propaganda to the enterprise, and an indirect affirmation and appreciation of the ability of enterprise managers. When a manager is praised by the media or society, it will stimulate the manager’s investment enthusiasm, further increase the degree of overconfidence, and make him more optimistic and positive about the investment environment and the future prospects of the project (Gao et al., 2021; Fan et al., 2022). When praised by society and news media, enterprise CEOs will be more confident, more optimistic about investment prospects and future returns, and thus make more and more aggressive investments (Brown et al., 2009). Under positive media reports, managers will further increase their overconfidence, pursue larger-scale expansion driven by higher interests, and are more likely to make irrational decisions that lead to overinvestment (Popa and Nedelea, 2022). Therefore, positive media reports cannot negatively regulate overinvestment caused by overconfidence, but rather aggravate overinvestment caused by managers’ overconfidence.

In addition, positive reports and publicity may form an “investment bubble” in the stock market, leading to rising stock prices and overvaluation of companies. In such a situation, the media makes enterprise financing more convenient through free and powerful publicity, and has ample cash flow (Wang, 2017; Tijani et al., 2021). At this time, managers will make more investment and lead to overinvestment. Moreover, when the media reports too much positively on the enterprise, the reputation mechanism will reduce the supervision of the enterprise by external stakeholders, relax the risk warning of the enterprise, and reduce the constraints and supervision of the investment behavior of the enterprise (Bai et al., 2019). As a result, managers lack reasonable and rational evaluation and consideration when making investment decisions, resulting in overinvestment of enterprises. To sum up, this paper proposes the hypothesis H2a:

Hypothesis H2a: Positive media reports can exacerbate overinvestment caused by managers’ overconfidence.

On the contrary, the negative reports of the media will generally affect the investment behavior of enterprises from three aspects. First, compared with positive media reports, negative reports are generally more well-founded and more credible. Therefore, negative reports usually have greater influence, and the market reaction caused by negative reports will be correspondingly stronger. Compared with positive reports, negative media reports can play a more important role in public opinion and supervision (Jin and Qin, 2021). Erena et al. (2022) and other studies found that the media reports and exposure of negative enterprise news will lead to a substantial decline in enterprise stock prices, affecting enterprise reputation and rating, and leading to a decline in enterprise investment capabilities (Li et al., 2018). Wang et al. (2022) deeply studied the relationship between enterprise performance and market response, and found that negative media reports can trigger a larger market response, thus playing the role of enterprise governance (Han et al., 2021). Second, negative media reports will draw widespread public attention. Especially under the trend of rapid development of mass media in recent years, negative reports will cause certain pressure on public opinion, which will lead to the high attention and key supervision of administrative and regulatory departments (Kottimukkalur, 2018). This gives enterprises stronger supervision, and it is easier, more accurate and timely to detect irrational behaviors and irregularities of enterprises. Under such pressure, negative media reports can improve social supervision, reduce overinvestment by enterprises, and achieve the purpose of enterprise governance. Third, media reports can have a significant impact on managers’ psychology. Negative press can damage a manager’s image and reputation. In order to restore their own image and enterprise reputation, managers will try their best to establish a positive image, invest in strict accordance with shareholders’ wishes and rational investment principles, reduce excessive investment behavior, and improve enterprise investment efficiency. On the other hand, the negative media reports on enterprises will undoubtedly cause a certain blow to managers’ psychology. The specific performance is that managers are more cautious when analyzing investment decisions, and will more objectively judge the value and risks of investment projects to avoid investment failures (Krulicky and Horak, 2021; Lu, 2022).

In addition, media reports of negative enterprise news will attract the attention and stricter supervision of both public investors and regulatory authorities in society. Such public opinion pressure will have a great negative impact on the career and future development of managers. Rossi et al. (2021) found that the supervision of the media has a strong binding force on managers, which will seriously affect the reputation and image of managers. Under the influence of the media, managers can effectively reduce the violations of managers’ self-interest trends. Rahayu et al. (2022) concluded that negative media reports will inhibit managers’ desire to satisfy their interests and play a role in enterprise governance. In summary, this paper proposes the following hypothesis H2b:

Hypothesis H2b: Negative media reports can inhibit overinvestment caused by managers’ overconfidence.

### Moderating effect of media reports under different marketization processes

China is currently under the institutional background of social market economic transformation with Chinese characteristics, which is a critical period of economic transformation. However, due to China’s vast territory and numerous provinces, the marketization process of each province and region is quite different (Durana et al., 2021). The marketization processes is a concentrated manifestation of the comprehensive environment of a region, which affects the activities and behaviors of different players in the market, and virtually supervises and restrains all players in the market (Kunjal et al., 2021; Akbar et al., 2022). As an important manifestation of the macro environment, the marketization processes will not only affect the governance role of the media, but also affect the behavior and decision-making of managers, thereby affecting the investment efficiency of enterprises (Kottimukkalur, 2018).

Positive media reports are not only difficult to achieve the role of enterprise governance, but also cannot suppress overinvestment caused by managers’ overconfidence, but will further aggravate managers’ overconfidence, which is more likely to lead to companies’ overinvestment. In areas where the marketization process is high, the market order and social system are relatively more complete, the degree of information asymmetry is lower, the mutual flow of information is more convenient, and the market is more transparent. The competition in the capital market is more intense, and there are more choices and opportunities for investors to invest in Rossi et al. (2021). The managers of enterprises will have higher pursuit and more urgent desire for promotion and reputation. At this time, the positive reports of the media will further expand, aggravate the overconfidence of managers, enhance the optimism of managers, stimulate managers to trigger their more enthusiastic investment enthusiasm, and then more easily lead managers to make excessive investment decision (Marjohan, 2021; Fan et al., 2022). In areas where the marketization process is low, investment opportunities are relatively limited, information asymmetry is high, market competition is not so intense, and the overall investment atmosphere and enthusiasm in the market are relatively low, and it is not easy to generate investment bubbles and follow-up investment. The aggravation of managers’ overconfidence by positive media reports is not very significant, and there may be a certain degree of lag (Suryani et al., 2021). Therefore, in an environment with a low degree of marketization, the impact of positive media reports on the degree of overconfidence of enterprise managers will be much smaller than that in areas with a high marketization process, and the aggravating effect of overinvestment caused by overconfidence is not as significant as that in areas with high marketization. In summary, this paper proposes the hypothesis H3a:

Hypothesis H3a: In regions with high marketization, positive media reports has a more pronounced effect on the relationship between managers’ overconfidence and overinvestment.

For negative media reports, it can play a positive role to improve enterprise governance. However, the marketization process itself can play a certain positive and governance role, which is a good supplement to the external governance and supervision mechanism. Lyan et al. (2021) concluded through research that there is no complementary role between the media and the marketization process, but an alternative relationship. In this society that is undergoing a market-oriented economic transition, in areas where the marketization process is high, the influence of the media will be weakened accordingly. That is to say, in areas with a low degree of marketization, the media, as a supplement of a governance mechanism, can make up for the insufficiency of the marketization process (Richardson, 2006). In regions with a high degree of marketization, the governance role of media reports will be weakened (Wang, 2017).

In areas where the process of marketization is relatively high, information transmission is relatively smooth, and the degree of information asymmetry is low. The information among all parties in the market is relatively transparent, and both managers and investors have multiple ways and means to obtain information and make decisions. Elberry and Hussainey (2020) also believes that in regions with high marketization, information flows smoothly between enterprises and external investors, and legal protection, competition mechanisms and other mechanisms can effectively reduce information asymmetry between the two parties. In addition, due to the relatively complete institutional norms and competition supervision mechanisms in the highly market-oriented regions, overconfidence prevails. Negative media reports have little effect on it, and it is difficult to suppress the excessive investment behavior caused by managers’ overconfidence (Shi et al., 2020; Miao, 2022). At this time, the role of media reports in enterprise governance was limited. In regions with a low level of marketization, the market capacity and capital are very limited, there are not many opportunities and choices in the market, and the competition and institutional mechanisms in the market are not perfect. Enterprise managers and external investors have limited access to information, and the cost is relatively high (Akbar et al., 2021). Moreover, the market supervision mechanism is not perfect, and the supervision of enterprises is not in place. In such an environment, negative media reports have a relatively large impact on society, greatly weakening managers’ self-confidence and investment enthusiasm, and in order to maintain their own reputation, it will reduce irrational decision-making and reduce excessive investment. At this time, the negative media reports will have a greater impact on enterprises and society, but can better play the role of enterprise governance (Ali et al., 2022; Yeoh and Hooy, 2022). To sum up, this paper proposes the hypothesis H3b:

Hypothesis H3b: Negative media reports have a stronger inhibitory effect on the relationship between managers’ overconfidence and overinvestment in regions with lower marketization.

The relationship structure between the research hypotheses in this paper is shown in Figure 2.

**FIGURE 2:** Research hypothesis relationship diagram.

## Research design

### Data sources

This paper selects all A-share listed companies in China from 2013 to 2021 as the research object, and based on this, the samples are screened as follows: (1) The financial data of listed companies in industries such as finance and insurance fluctuates greatly, which will affect the research hypotheses of this paper, so industry samples such as finance and insurance are excluded. (2) The lack and abnormality of relevant data of the enterprise will make it impossible to reflect the real situation of the enterprise normally, so the samples with missing data and abnormal financial data are excluded. (3) There is a certain suspicion of fraud in the relevant data of ST company, so the sample of listed companies that were ST was excluded during the research period. In addition, in order to alleviate the influence of extreme values in the sample on the empirical results, the Winsorize extreme value adjustment is performed on the sample at the 1 and 99% levels to eliminate the influence of extreme values on this study. Through elimination and screening, the balanced panel data of 6,012 companies are finally obtained as research samples. Likewise, the methodology of this study allows the study to be replicated in numerous countries such as the United States or Europe.

The variable data used in this article are mainly from the China Stock Market and Accounting Research Database (CSMAR) and China National Knowledge Infrastructure (CNKI): (1) The media reports data is obtained through the subject search of the full name and abbreviation of the listed company by the eight major newspapers and magazines in the “Full-text Database of Important Chinese Newspapers” of CNKI with the help of Python software. (2) Data on other variables are mainly collected through the CSMAR database. All data were processed and empirically analyzed using STATA15.0 software.

### Variable selection

#### Predicted variables

Richardson (2006) is currently the most widely used and effective model for measuring investment efficiency. The principle of the model is: under the premise of considering the factors that affect the investment amount, the difference between the expected and actual investment amount of the enterprise is used to represent the investment efficiency of the enterprise. This model cannot only conveniently distinguish inefficient investment, but also measure the intensity of inefficient investment, and does not need to rely on the Tobin Q value of enterprises, and it is also applicable in Chinese’s capital market. Based on this, this paper uses the Richardson (2006) model to measure overinvestment. This paper calculates the company’s investment efficiency to measure the company’s overinvestment. The residual ε_*it*_ is used to represent the inefficient investment of the enterprise, and only the samples with the residual ε_*it*_ greater than 0 are retained.


Investit=α0+αG1rowthi,t-1+α2Levi,t-1+α3Cashi,t-1+αA4gei,t-1+αS5izei,t-1+αR6eti,t-1+αI7nvesti,t-1+∑Industry+∑Year+εit

#### Explanatory variables

This paper argues that the use of personal background characteristics to measure managers’ overconfidence is a relative value. Methods are more rational, personal characteristics are more objective, and uncertainty and subjectivity are avoided. Therefore, this paper uses gender, dual-job integration, age and educational background to construct a comprehensive indicator to measure managers’ overconfidence:

##### Sexsorce

Byrnes et al. (1999) found that compared with women, men are more radical, they are too firm in their own judgments and choices, and it is difficult to listen to others’ opinions, and there is a more serious overconfidence mentality. Clifton and Gill (1994) specifically studied the influence of gender on self-confidence psychology. The results showed that women were far less confident than men, and women were more conservative and underestimated their abilities.

##### Agescore

With the growth of age, people’s knowledge and experience will become more and more rich, and their decisions will generally become more mature and rational. Lyan et al. (2021) found that, after experiencing some failures, older managers will learn from experience and continuously improve their judgment and decision-making ability, thereby reducing their overconfidence and irrational mentality. Especially in investment projects, they are more cautious and prudent in order to avoid risks, and their degree of overconfidence is much lower than that of younger managers (Greene, 2006). Therefore, the text argues that managers with younger age indicators are more prone to overconfidence and have higher levels. In this paper, the age indicator is defined as the ratio of the difference between the maximum and observed age in all samples to the difference between the maximum and minimum values in all samples. The higher the score, the higher the degree of overconfidence.


$$agescore=\frac{\max\left(age\right)-age}{\max\left(age\right)-\min\left(age\right)}$$

##### Degreescore

People with higher education have the capital to think they have higher ability and richer investment experience. The research of Schrand and Zechman (2011) shows that the higher the education level, the more confident you will be, who think you have a higher ability, tend to overestimate your true level, and firmly believe that your judgment and choice are correct. Therefore, this paper believes that managers with higher education are prone to overconfidence. The higher the education, the stronger the sense of superiority and the higher the degree of overconfidence. Therefore, when the manager has a bachelor’s degree or above, the education index takes the value of 1, otherwise it is 0.

##### Posiscore

*Posiscore* refers to a manager being awarded two key positions at the same time by a company. People with dual positions and high positions are more confident, further exacerbating the level of managers’ overconfidence. Managers see this as an affirmation and appreciation of their own abilities, which further increases their confidence in decision-making (Schrand and Zechman, 2011). Therefore, this paper believes that if a manager holds two positions, it will be more prone to overconfidence, that is, if the manager has two positions, the indicator takes a value of 1, otherwise it is 0.

Overconfidence (***OC***): The degree of managers’ overconfidence is comprehensively measured and reflected by personal characteristics. This paper sums up the above four personal characteristics to their arithmetic average, and uses the final score as a measure of managers’ overconfidence.


$$OC=\frac{sexscore+agescore+degreescore+posiscore}{4}$$

#### Moderating variables

##### Media

At this stage, the media mainly include newspapers and magazines, online media and self-media. Compared with newspapers and magazines, online media and self-media are greatly affected by other factors, and the voices are complex and changeable, their objectivity and credibility are low, and their credibility is not as good as that of newspapers. On the other hand, it is difficult to obtain and collect information on online media and self-media, and it is difficult to do a comprehensive arrangement. Therefore, this paper selects the number of newspapers, magazines and self-media reports on enterprises as the measure of media reports.

This paper selects the eight most authoritative and influential mainstream financial newspapers in China as the source of media reports. The eight newspapers are “China Securities Journal,” “Securities Times,” “Shanghai Securities News,” “Securities Daily,” “China Business News,” “twenty-first Century Business Herald,” “First Financial Daily” and “Economic Observer.” The reason for choosing these eight newspapers is that the first four newspapers are official media specially and strictly stipulated by the China Securities Regulatory Commission, and they are policy-oriented media with sufficient authority. The last four newspapers are relatively authoritative media organizations in Chinese’s securities industry and even in the entire market, with very large market influence and circulation. Therefore, choosing these eight newspapers as the source of media reports has sufficient authority and persuasion.

This paper measures media reports by the natural logarithm of “1 ++++ the number of media reports”, defined as *Media*. In order to further study the different influences and roles of positive and negative media reports, media reports need to be divided into positive and negative reports according to their content. Since there is no uniform and standard division on how to divide positive and negative reports, this paper distinguishes positive media reports (*P*_*Media*_) and negative media reports (*N*_*Media*_) according to the content of the report by reading each report and according to the emotional color. When statements such as “tax evasion, shady, illegal, corrupt, fraud” appear in the report, it is a negative report. When statements such as “optimize, improve, perfect” appear in the report, it is a positive report. In order to prevent endogeneity, the data reported by the media in this paper is measured by the number of media reports with a lag period of one period, that is, period *t*-1. The specific measurement methods of media reports variables are as follows:


$$\begin{array}{ccc} P_{Media} & = & \ln\left(1+Number\;of\;positive\;media\;reports\right)\\ N_{Media} & = & \ln\left(1+Number\;of\;negative\;media\;reports\right) \end{array}$$

#### Control variables

(1) Enterprise age (*Age*)

*Age* represents the age of the company’s listing. The shorter the company’s listing period, the less perfect the internal governance mechanism, and the more likely it is that irrational behaviors such as overinvestment will occur.

(2) Growth ability (*Growth*)

The higher the growth ability (*Growth*) of the enterprise, the more funds it accumulates and the more investment opportunities, the more capital and opportunities for overconfident managers to use sufficient free cash flow to invest, and thus more prone to overinvestment behavior. This paper uses the “main business income growth rate” to measure the growth ability of enterprises.

(3) Marketization process (*Market*)

*Market* is a process of economic transition, involving a series of social, institutional, economic, political and other transformations, and it is difficult to measure it with a single indicator. This paper deeply explores the characteristics of China’s marketization process, and constructs a comprehensive index through principal component analysis, namely, the marketization process index. The marketization process index can generally reflect the degree of marketization and differences in various provinces and regions, and is currently the most reasonable and perfect method to measure China’s marketization process. The higher the regional marketization index, the faster the marketization process in the region, the higher the marketization level, the more perfect the laws and competition mechanisms, and the less government administrative intervention. This paper sets “*Market”* as a dummy variable. When the marketization process index in the region is higher than the average index, the value is 1, otherwise it is 0.

(4) Equity concentration (*Top* 1)

*Top* 1 is the ratio of the number of shares held by the largest shareholder to the total number of shares. The greater the voice of the largest shareholder, the stronger the control over decision-making, the more likely it is to check and balance the irrational behavior of managers, thereby reducing the excessive investment of enterprises. However, when the largest shareholder also has overconfidence, it may further exacerbate the company’s overinvestment. This paper uses “the ratio of the number of shares held by the largest shareholder to the number of all ordinary shares” to measure the ownership concentration.

(5) Enterprise size (*Size*)

The size of the enterprise is the embodiment of the comprehensive strength of the enterprise. In general, the larger the enterprise scale, the more investment opportunities the enterprise has, and the managers have a stronger sense of superiority and more overconfidence, believing that the enterprise is strong enough to withstand any risks. In this paper, the natural logarithm of “total assets” is used to measure the size of the enterprise.

(6) Return on Equity (*Roe*)

The higher the *Roe* of an enterprise, the better the overall vitality of the enterprise and the better the operating income. Managers will also have a more optimistic attitude toward the development prospects of the company, and will be more prone to overinvestment. This paper uses the ratio of net profit to average shareholders’ equity of the enterprise to measure.

(7) *Industry*

Industry is a dummy variable that controls the influence of different industry factors. The media’s attention and reports of different industries are different, so the number of media reports of companies in different industries is also quite different. This paper divides the sample enterprises into 18 industries, so this paper sets 17 industry dummy variables.

(8) Annual (*Year*)

*Year* is a dummy variable to control the influence of different year factors. The number of times the media reports on companies varies in different years. This paper takes the listed companies from 2013 to 2021 as a sample, with a total of 9 years of data, so a total of 8 annual dummy variables are set.

In summary, the selection and definitions of all variables in this paper are shown in Table 1.

**TABLE 1:** Variable definition table.

Type	Name	Symbol	Definition
Predicted variables	Overinvestment	***Overinv***	Calculated using the Richardson model
Explanatory variables	Managers’ overconfidence	***OC***	Arithmetic mean of managers’ personal characteristics
Moderating variables	Positive media reports	***P*_*Media*_**	ln(1+Number of positive media reports)
	Negative media reports	***N*_*Media*_**	ln(1+Number of negative media reports)
Control variables	Equity concentration	***Top* 1**	Shareholding ratio of the largest shareholder
	Enterprise age	***Age***	The company’s listing period
	Return on equity	***Roe***	Net profit/Average Shareholders’ equity
	Enterprise growth	***Growth***	Growth rate of current operating income
	Enterprise size	***Size***	The natural logarithm of the company’s total assets
	Marketization	***Market***	Marketization index of each province. 1 for above average, 0 otherwise.
	Industry	***Industry***	The sample involves 18 industries and 17 dummy variables are set
	Year	***Year***	The sample involves 9 years, and 8 dummy variables are set

### Model design

This study uses China’s 2013–2021 A-share listed companies in Shanghai and Shenzhen as a sample to explore the relationship between managers’ overconfidence, positive and negative media reports, and overinvestment. In order to verify the hypotheses of this paper, the following regression equation is established to test the relevant hypotheses proposed in this paper.

Research on the impact of managers’ overconfidence on enterprise overinvestment:


$$Overinvit=\beta_{0}+\beta_{1}OC_{it}+\sum \gamma_{i}Controls+\varepsilon_{it}$$

To study the moderating effect of positive and negative media reports on managers’ overconfidence and enterprise overinvestment relationship and the heterogeneity analysis of marketization process:


$$\begin{array}{ccc} Overinvit=\beta_{0}+\beta_{1}OC_{it}+\beta_{2}OC\times P_{Media}+\beta_{3}P_{Media}+\sum \gamma_{i}Controls+\varepsilon_{it} & & \\ Overinvit=\beta_{0}+\beta_{1}OC_{it}+\beta_{2}OC\times N_{Media}+\beta_{3}N_{Media}+\sum \gamma_{i}Controls+\varepsilon_{it} & & \end{array}$$

## Empirical test and result analysis

### Descriptive statistics

This paper collects and organizes the data of all A-share listed companies from 2013 to 2021. After excluding unqualified samples, a total of 6,012 observations are obtained. In order to reduce the influence of abnormal values on the results, the data were processed with 1% unilateral or bilateral Winsorize. The descriptive statistical results are shown in Table 2.

**TABLE 2:** Descriptive statistics.

Variable name	*Mean*	*Std.*	*Min*	*Max*
***Overinv***	0.058	0.076	0.0004	0.42
***OC***	0.659	0.151	0.026	0.996
***P*_*Media*_**	1.058	0.949	0	6.103
***N*_*Media*_**	1.050	0.977	0	6.304
***Top* 1**	0.339	0.145	0.0880	0.75
***Growth***	0.442	1.279	–0.723	2.018
***Size***	22.430	1.246	19.66	26.06
***Age***	17.810	5.707	4	31
***Roe***	0.063	0.122	–0.819	0.313
***Market***	0.568	0.495	0	1

From the descriptive statistical results in Table 2, the *Mean* of *Overinv* is 0.058, the *Std.* is 0.076, the *Max* is 0.42, and the *Min* is 0.0004. The phenomenon of overinvestment is common, but there are certain differences in its degree; the *Max* is much higher than *Mean*, that is, the current degree of overinvestment of listed companies is relatively serious.

The *Mean* of the *OC* is 0.659, indicating that 65.9% of the enterprise managers in the research sample enterprises are overconfident. The *Max* of overconfidence is 0.996, the *Min* is 0.026, and the *Std.* is 0.151, which indicates that the severity of overconfidence among different managers is quite different.

The *Mean* of *P*_*Media*_ is 1.058, the *Max* is 6.103, and the *Min* is 0, indicating that the positive media reports of enterprises varies greatly. Some companies have been positively promoted by the media many times, while some companies have never been positively reported by the media. The *Mean* of *N*_*Media*_ is 1.050, the *Max* is 6.304, and the *Min* is 0, indicating that there are also great differences in the negative media reports of enterprises. Some companies have no negative reports, while others are frequently negatively reported by the media.

The *Mean* of *Top* 1 is 0.339, the *Max* is 0.75, and the *Min* is 0.0880, indicating that the difference in *Top* 1 between different companies is very significant. The *Mean* of *Growth* is 0.442, the *Max* is 9.018, the *Min* is -0.723, and the *Std.* is 1.279, indicating that the sample covers enterprises with various growth ability levels and has a wide range. The *Mean* of *Size* is 22.43, the *Max* is 26.06, and the *Min* is 19.66. The *Mean* of *Age* is 17.81. The longest listed company is 31 years, and the shortest is 4 years. It is more meaningful to study the behavior of companies with longer listing years. The *Max* of the *Roe* of the enterprise is 0.313, the *Min* is -0.819, and the *Mean* is 0.063, indicating that the income of the sample enterprises is quite different. The *Market* is used as a dummy variable with a mean value of 0.568.

### Correlation analysis

Before the regression analysis, this paper uses the Pearson coefficient test to analyze the correlation of each variable, and preliminarily judges whether there is a correlation between overconfidence and overinvestment, positive and negative media reports and overinvestment. The results are shown in Table 3.

**TABLE 3:** Correlation coefficient test table.

Variables	*Overinv*	*OC*	*P*_*Media*_	*N*_*Media*_	*Top* 1	*Growth*	*Size*	*Age*	*Roe*	*Market*
***Overinv***	1.000									
***OC***	0.050***	1.000								
***P*_*Media*_**	0.046***	–0.006	1.000							
***N*_*Media*_**	−0.023**	–0.013	0.737***	1.000						
***Top* 1**	–0.011	−0.029**	0.078***	0.081***	1.000					
***Growth***	0.085***	0.014	0.024**	0.034***	0.033***	1.000				
***Size***	−0.052***	−0.062***	0.350***	0.334***	0.180***	0.049***	1.000			
***Age***	−0.106***	−0.094***	−0.117***	−0.071***	−0.085***	0.084***	0.221***	1.000		
***Roe***	0.067***	−0.027**	0.134***	0.065***	0.129***	0.047***	0.114***	−0.045***	1.000	
***Market***	–0.003	0.080***	−0.097***	−0.091***	0.034***	0.016	−0.018*	−0.020*	0.015	1.000

***p < 0.01, **p < 0.05, *p < 0.1.

From the results in Table 3, it can be concluded that the relationship between *OC* and *Overinv* is significantly positive at the 1% level. That is, managers’ overconfidence will lead to overinvestment, which is consistent with the previous hypothesis H1. The relationship between *P*_*Media*_ and *Overinv* is significantly positive at the 1% level, and positive media reports will aggravate enterprise overinvestment. The relationship between *N*_*Media*_ and *Overinv* is significantly negative at the 5% level. It shows that the negative media reports can negatively regulate the excessive investment of enterprises, improve enterprise governance to a certain extent, and play a role in raising the level of investment. The results are in line with the previous hypotheses of H2a and H2b.

*Top* 1 is negatively correlated with overinvestment, but not significant. The higher the shareholding ratio of the largest shareholder, can reduce its irrational behavior to a certain extent and reduce the excessive investment of enterprises, but there is no completely significant correlation between these two variables. The *Growth* and overinvestment are significantly positively correlated at the level of 1%, that is, the stronger the *Growth*, the more capital there is for investment activities. *Size* and overinvestment are significantly negatively correlated at the 1% level. The larger the *Size*, the more comprehensive the assessment will be carried out before the investment for risk management and control, so as to alleviate overinvestment. *Age* is significantly negatively correlated with overinvestment at the 1% level. The longer the *Age*, the more inclined the company will be to stabilize its market position and consolidate its market share, prefer the strategy of seeking progress while maintaining stability, and be less likely to overinvestment. *Roe* is positively related to overinvestment, but not significantly. Higher enterprise performance and fewer financing constraints may encourage managers to overinvestment with ample cash flow.

From the results of the correlation test data, the relationship between the variables studied in this paper is basically in line with the expected expectations. This paper will further analyze and test all the hypotheses in depth in the empirical testing section.

### Multiple regression analysis

This paper divides the sample into three sections for research. The first section tests Hypothesis H1 and studies the effect of managers’ overconfidence on overinvestment. Section “Literature review” verifies hypotheses H2a and H2b, introduces media reports as a moderating variable, and studies whether positive or negative media reports has moderating effects on managers’ overconfidence-induced overinvestment. Section “Research hypothesis” verifies hypotheses H3a and H3b, and studies the moderating effect of media reports under different marketization processes.

#### Impact of managers’ overconfidence on enterprise overinvestment

In this paper, the regression results of hypothesis H1 through empirical testing are shown in Table 4. In the regression process, industry and year were controlled.

**TABLE 4:** Regression results of managers’ overconfidence on overinvestment.

Variables	Coefficient	*T*-value	VIF
***OC***	0.0179***	2.8125	1.258
***Top* 1**	−0.0010**	−0.1418	1.024
***Growth***	0.0078***	8.9484	1.172
***Size***	–0.0004	−0.4089	1.023
***Age***	−0.0007***	−3.7375	1.087
***Roe***	0.0389***	4.5271	1.402
***Market***	0.0020*	0.9479	1.128
***Industry***		Control	
***Year***		Control	
***Constant term***	0.0345	1.3260	
***F-value***		4.5	
***Sig.***		0.0000***	
***Durbin-Watson***		1.7325	
***Number of samples***		6,012	
***Adj.R* ^2^**		0.271	

***p < 0.01, **p < 0.05, *p < 0.1, the same below.

##### Goodness of fit, F-test, VIF test analysis

According to Table 4, the *Adj.R*^2^ is 0.271, indicating that all explanatory variables in the model explain 27.10% of the *Overinv* of the predicted variable, and the model has a good goodness of fit. The *F-value* is 4.5 and the *Sig.* is 0.0000, indicating that the model is statistically significant. The VIF of all variables did not exceed 2, indicating that there was no multicollinearity among the variables. The *Durbin-Watson* is 1.7325, which is small, indicating that the random error term does not have autocorrelation.

##### Significant analysis

It can be seen from Table 4 that *OC* and *Overinv* have a significant positive correlation at the 1% confidence level. Looking at the control variables, *Growth* and *Roe* are significantly positively correlated with *Overinv*, and *Age* is significantly negatively correlated with *Overinv*.

##### Analysis of test results

From Table 4, it can be concluded that the regression coefficient of (*OC* and *Overinv* is 0.0170, which is significantly positive at the 1% level, indicating that managers’ overconfidence will directly lead to overinvestment of enterprises. When managers are overconfident, they have a strong sense of superiority, trust their own judgments too much, are optimistic about the future rate of return of the project, and have difficulty listening to the opinions of others. Driven by their own promotion and interests, managers will prefer to invest in expansion, easily choose non-quality projects, make excessive investment, and weaken the value of the enterprise. Through the above test and analysis, it can be concluded that there is a positive correlation between managers’ overconfidence and overinvestment, which verifies the establishment of hypothesis H1: managers’ overconfidence will lead to overinvestment.

In terms of control variables, the regression coefficient between Top 1 and overinvestment is -0.001, but it is not significant. It shows that the higher the shareholding of the largest shareholder, it is only possible to supervise and balance the managers and reduce excessive investment, but it cannot realize the role of enterprise governance. The regression coefficient between the *Growth* and overinvestment is 0.0078, which is significantly correlated at the 1% confidence interval. It shows that the higher the growth ability of the company, the faster the growth of the company’s operating income and the better the performance, which will prompt the company to use sufficient cash flow for investment, thereby increasing the possibility of the company’s overinvestment. The regression coefficient between *Size* and overinvestment is -0.0004, but not significant. It shows that the larger the size of the enterprise, it may reduce the overinvestment of the enterprise, but the size of the enterprise does not have a direct and significant impact on whether the enterprise is overinvested. The regression coefficient between *Age* and overinvestment is -0.0007, and there is a significant correlation within the 1% confidence interval. It shows that the younger the enterprise is, the more immature and imperfect the relevant internal regulatory checks and balances are, and the enterprise is in the growth stage and prefers to expand, the more likely it is to make over-investment. On the contrary, the longer the company has been listed, the more conservative and stable the enterprise strategy will be, and there will be less overinvestment. The regression coefficient between *Roe* and overinvestment is 0.0389 and is significantly correlated within the 1% confidence interval. When the ratio between enterprise net profit and shareholders’ equity increases by 1 percentage point, enterprise overinvestment will increase by 0.0389 percentage points. That is, the better the performance of the enterprise, the more likely it will lead to further overinvestment of the enterprise.

#### Moderating effect of media reports on managers’ overconfidence and overinvestment

This section further explores how media reports influence and moderate the overinvestment behaviors of companies caused by managers’ overconfidence under different emotional colors. The regression results are shown in Table 5.

**TABLE 5:** Regression results of the moderating effect of positive and negative media reports.

Variables	Coefficient	*T*-value	VIF	Coefficient	*T*-value	VIF
***OC***	0.0133***	–1.5475	1.0315	0.0369***	4.8131	1.0296
***P*_*Media*_**	−0.0186***	–4.4936	1.2416			
***P_*Media*_ × OC***	0.0354***	5.3893	1.3872			
***N*_*Media*_**				0.0101***	3.0776	1.0243
***N_*Media*_ × OC***				−0.0244***	–4.3273	1.1378
***Top* 1**	0.0007	0.0965	1.0582	–0.003	–0.4251	1.0582
***Growth***	0.0078***	8.9947	1.3736	0.0078***	9.0122	1.3736
***Sise***	–0.0012	–1.1716	1.0583	0.0006	0.6345	1.0583
***Age***	−0.0007***	–3.6443	1.1254	−0.0007***	–3.7318	1.1254
***Roe***	0.0373***	4.3308	1.3127	0.0393***	4.5786	1.3127
***Market***	0.0040*	1.8852	1.4139	0.0002	0.0757	1.4139
***Industry***		Control			Control	
***Year***		Control			Control	
***Constant term***	0.0668**	2.4479		0.0108	0.4002	
***F-value***		17.89			9.84	
***Sig.***		0.0000***			0.0000***	
***Durbin-Watson***		1.2376			1.8356	
***Number of samples***		6,012			6,012	
***Adj.R* ^2^**		0.209			0.194	

***p < 0.01, **p < 0.05, *p < 0.1.

##### Goodness of fit, F-test, VIF test analysis

Regarding the regression of the moderating effect of positive media reports, as shown in Table 5, the *Adj.R*^2^ was 0.209. It shows that the variable in the model explains the *Overinv* of the predicted variable is 20.90%, which has a good goodness of fit. The *F-value* is 17.89 and the *Sig.* is 0.0000, indicating that the model has significant statistical significance. The VIFs of all variables were around 1.0, indicating that there was no multicollinearity among the variables. The *Durbin-Watson* is 1.2376, indicating that there is no autocorrelation in the random error term.

Regarding the regression of negative media reports and overinvestment, according to Table 5, the *Adj.R*^2^ is 0.194. It shows that the variables in the model explain the degree of *Overinv* of the predicted variable is 19.4%, which has a good goodness of fit. The *F-value* was 9.84 and the *Sig.* was 0.0000, indicating that the model was statistically significant. The VIFs of all variables were around 1.0, indicating that there was no multicollinearity among the variables. The *Durbin-Watson* is 1.8356, indicating that there is no autocorrelation in the random error term.

##### Significant analysis

From Table 5, it can be seen that the media positive reporting interaction term (*P_*Media*_* × *OC*) and overinvestment are significantly positive at the 1% confidence level. The *Growth, Roe* and *Market* have a significant positive correlation with overinvestment. *Age* has a significant negative correlation with overinvestment. The relationship between *Size* and *Top* 1 and *Overinv* is not significant. While the negative media reports interaction term (*N_*Media*_* × *OC*) and overinvestment are significantly negative at the 1% confidence level, the regression results for the control variable and overinvestment are similar to the previous regression results.

##### Analysis of test results

From the results in Table 5, it can be seen that the regression coefficient between the positive media reports item (*P_*Media*_* × *OC*) and the *Overinv* is 0.0354, and there is a significant positive correlation at the 1% confidence level. The regression coefficient between the negative media reports item (*N_*Media*_* × *OC*) and the *Overinv* is −0.0244, which is significantly negatively correlated at the 1% level. The above results show that positive media reports will aggravate managers’ overconfidence, which will make enterprise managers optimistic about the future returns and prospects of investment projects, ignoring investment projects and market risks, and further lead to excessive investment behavior. The negative reports and exposure of the media to the enterprise will cause a certain blow to the managers, reduce their overconfidence psychology, and also have a certain impact on the reputation and image of the enterprise. For the sake of their own development and enterprise image, managers will be more cautious and prudent in investment, and evaluate the risks of investment projects more comprehensively and accurately. Managers prove to investors the ability of managers and the good prospects of enterprises through correct investment behaviors and performance, thereby reducing the excessive investment behaviors of enterprises caused by managers’ overconfidence, and effectively realizing enterprise governance. The above analysis verifies the hypothesis H2a and H2b, respectively.

#### Moderating effect of media reports under different marketization processes

At present, China is in the critical stage of market-oriented economic transformation. Different market-oriented processes have different impacts on the development of enterprises. In addition to Chinese’s unique national conditions, the level of regional marketization varies greatly. Under different economic and legal environments, media reports play different roles. In order to more accurately analyze how media reports affect the overinvestment caused by managers’ overconfidence under different marketization processes. This paper divides the samples into high and low groups according to the marketization process, and divides the sample enterprises into high marketization and low marketization for analysis.

First, study the moderating effect of media positive reports on overconfidence and overinvestment under different marketization processes. The regression results are shown in Table 6.

**TABLE 6:** Regression results of positive media reports under different marketization processes.

	Low marketization			High marketization		
Variables	Coefficient	*T*-value	VIF	Coefficient	*T*-value	VIF
***OC***	0.0120***	0.8437	1.3178	0.0331***	–3.0226	1.1472
***P*_*Media*_**	0.0015***	0.2422	1.2012	−0.0400***	–6.8745	1.9134
***P_*Media*_ × OC***	0.0005	–0.0485	1.7213	0.0691***	7.8372	1.1165
***Top* 1**	0.0028	0.260	1.3421	0.0016	0.1708	1.2465
***Growth***	0.0107***	7.7314	1.2984	0.0063***	5.5924	1.2312
***Sise***	0.0012	0.7457	1.6597	−0.0024*	–1.7952	1.0312
***Age***	−0.0007**	–2.0448	1.2165	−0.0008***	–3.2662	1.1432
***Roe***	0.0502***	3.7756	1.0159	0.0308***	2.6748	1.2169
***Industry***		Control			Control	
***Year***		Control			Control	
***Constant term***	–0.0061	–0.1616		0.1291*	1.6644	
***F-value***		22.34			18.02	
***Sig.***		0.0000***			0.0000***	
***Durbin-Watson***		1.2578			1.1895	
***Number of samples***		2,534			3,478	
***Adj.R* ^2^**		0.216			0.190	

***p < 0.01, **p < 0.05, *p < 0.1.

##### Goodness of fit, F test, VIF test analysis

According to Table 6, it can be concluded that in the sample group with a high degree of marketization, the *Adj.R*^2^ after regression is 0.190, and the *Adj.R*^2^ after regression in the sample group with a low degree of marketization is 0.216. It can be seen that the goodness of fit of the two sets of results is good and acceptable. The *F-values* were 18.02 and 22.34, respectively, and the *Sig.* were both 0.0000, indicating that the models were all statistically significant. None of the variables VIF exceeds 2, indicating that there is no multicollinearity among the variables. The *Durbin-Watson* are 1.1895 and 1.2578, respectively, indicating that there is no autocorrelation in the random error term.

##### Significant analysis

In regions with a high degree of marketization, the positive media reports item (*P_*Media*_* × *OC*) is significantly positively correlated with *Overinv*. *Growth, Roe* and *Overinv* are significantly positively correlated. *Age* has a significant negative correlation with *Overinv*. There was no significant relationship between the other control variables overinvestment.

##### Analysis of test results

From the data analysis in Table 6, in regions with low degree of marketization, the regression coefficient between positive media reports (*P_*Media*_* × *OC*) and *Overinv* is 0.0005, but it is not significant. In regions with a high degree of marketization, the regression coefficient between the positive media reports item (*P_*Media*_* × *OC*) and the *Overinv* is 0.0691, and it is significantly correlated at the 1% level. This shows that in regions with a high degree of marketization, market competition is more intense, investment opportunities are more numerous, managers’ pursuit of self-promotion and reputation is more urgent, and utilitarian psychology is more serious. In such an environment, positive media propaganda and reports will put more emphasis on managers’ overconfidence, which will lead to companies’ overinvestment behavior. On the contrary, in regions with a low degree of marketization, the market competition is not fierce and the projects that can be invested are limited. At this time, the positive media reports may have a relatively weak effect on managers’ psychology, or there may be a certain lag, and the impact on overinvestment caused by overconfidence is relatively small. The above results and analysis verify the above hypothesis H3a: in regions with high marketization, positive media reports have a more pronounced effect on the relationship between managers’ overconfidence and overinvestment.

Table 7 shows the moderating effect of negative media reports under the heterogeneity of the marketization process.

**TABLE 7:** Regression results of negative media reports under different marketization processes.

	Low marketization			High marketization		
Variables	Coefficient	*T*-value	VIF	Coefficient	*T*-value	VIF
***OC***	0.0786***	5.7165	1.0125	0.0255***	2.6732	1.0237
***N*_*Media*_**	0.0346***	5.8111	1.0365	–0.0003	–0.0832	1.6254
***N_*Media*_ × OC***	−0.0675***	–6.9055	1.3485	–0.0039	–0.5312	1.3485
***Top* 1**	–0.0005	–0.0462	1.1765	–0.0022	–0.2401	1.0265
***Growth***	0.0105***	7.680	1.4954	0.0063***	5.5963	1.1396
***Sise***	0.0030*	1.9242	1.0397	–0.0007	–0.5349	1.0358
***Age***	−0.0006*	–1.928	1.0575	−0.0008***	–3.4359	1.0954
***Roe***	0.0513***	3.9216	1.5469	0.0329***	2.8377	1.5279
***Industry***		Control			Control	
***Year***		Control			Control	
***Constant term***	−0.0688*	–1.8495		0.0602	0.7712	
***F-value***		23.72			6.29	
***Sig.***		0.0000***			0.0000***	
***Durbin-Watson***		1.2508			1.0685	
***Number of samples***		2,534			3,478	
***Adj.R* ^2^**		0.292			0.270	

***p < 0.01, *p < 0.1.

##### Goodness of fit, F test, VIF test analysis

According to Table 7, it can be concluded that in the sample group with a high degree of marketization, the *Adj.R*^2^ after regression is 0.270, and the *Adj.R*^2^ after regression in the sample group with a low degree of marketization is 0.292. It can be seen that the goodness of fit of the two sets of results is good and acceptable. The *F-value* were 6.29 and 23.72, respectively, and the *Sig* were both 0.0000, indicating that the models were all statistically significant. All variables VIF did not exceed 2, indicating that there was no multicollinearity among the variables. The *Durbin-Watson* are 1.0685 and 1.2508, respectively, indicating that there is no autocorrelation in the random error term.

##### Significant analysis

In regions with a high degree of marketization, the crossover term (*N_*Media*_* × *OC*) is negatively correlated with *Overinv*, but it is not significant. For the control variables, *Growth, Roe* and *Overinv* are significantly positively correlated, and *Age* is significantly negatively correlated with *Overinv*. There was no significant relationship between the other control variables overinvestment. In regions with low marketization, the crossover term (*N_*Media*_* × *OC*) and overinvestment (*Overinv*) are significantly negatively correlated at the 1% level. For the control variables, except that the *Age* has a significant negative correlation with the *Overinv*, the regression results of other control variables are similar to the above results, and will not be repeated here.

##### Analysis of test results

From the data analysis in Table 7, in low marketization regions, the regression coefficient between the negative media reports term (*N_*Media*_* × *OC*) and overinvestment is -0.0675, and it is significantly correlated at the 1% confidence level. In high marketization regions, the regression coefficient between the negative media reports term (*N_*Media*_* × *OC*) and overinvestment is -0.0039, but it is not significant. This shows that in regions with a high degree of marketization, legal, competition, and enterprise checks and balances are more complete and sound, which alleviates information asymmetry and agency costs between companies and the outside world, and the media plays a very limited role. Managers still underestimate the investment risks of projects, thereby reducing the governance effect of negative media reports. For areas with a low degree of marketization, information is relatively blocked, various legal mechanisms in the society are not perfect, and the internal checks and balances and supervision mechanisms of enterprises are not perfect. The information asymmetry and agency conflict in the enterprise will be more serious, and the government and other administrative departments will intervene relatively more, and the negative exposure of the media will have a greater impact on the enterprise and society. Negative media reports have a strong weakening effect on managers’ overconfidence, which can more effectively negatively regulate the over-investment caused by managers’ overconfidence, and can play a role in enterprise governance. This further verifies the view of many scholars that “media governance and marketization are an alternative relationship, not a complementary relationship.” The above results and analysis verify the above hypothesis H3b: in regions with a lower degree of marketization, negative media reports has a stronger inhibitory effect on the relationship between managers’ overconfidence and overinvestment.

In order to be able to see the regression results of all hypotheses in this paper more intuitively, this paper summarizes all the empirical test results, as shown in Table 8.

**TABLE 8:** Summary of variable regression results.

Hypothesis	Variable relationship		Salience	Empirical results
H1	Managers’ overconfidence leads to overinvestment		Significantly positive	Hypothesis H1 holds.
H2a	Moderating effect of positive media reports		Significantly positive	Hypothesis H2a holds.
H2b	Moderating effect of negative media reports		Significantly negative	Hypothesis H2b holds.
H3a	Moderating effect of positive media reports	High marketization	Significantly positive	Hypothesis H3a holds.
		Low marketization	Not significantly	
H3b	Moderating effect of negative media reports	High marketization	Not significantly	Hypothesis H3b holds.
		Low marketization	Significantly negative	

### Robustness check

Overconfident managers will psychologically believe that they have higher abilities and talents, which can bring more benefits to the company. Managers will have higher remuneration requirements in real enterprises, and the higher the remuneration paid to managers, the more overconfident managers will be (Luo and Ye, 2015). Therefore, this paper replaces the measure of overconfidence with relative compensation to conduct a robustness test, that is, “the sum of the top three CEO compensation” divided by “the sum of all compensation,” and the ratio is compared with the sample median. If the ratio is greater than the median, it is considered that the manager is overconfident, and the overconfidence (*OC*1) value is 1 at this time, otherwise it is 0.

Expanding the scope of newspapers and magazines to reflect the comprehensiveness of media reports is also to avoid bias in selecting samples (Jiang et al., 2009). In the selection of samples, in addition to the eight authoritative media magazines, other 500 other media newspapers and periodicals in the CNKI database were further selected, including important central newspapers, financial and economic newspapers, local morning newspapers, evening newspapers, and express news. The positive and negative reports are also distinguished according to their emotional colors, and the natural logarithms are recorded as *P*_*Media*_2 and *N*_*Media*_2, respectively.

In this paper, the above models are re-regressed after changing the measurement methods of variables. The specific regression results are as follows.

(1) Robustness test of the impact of managers’ overconfidence on enterprise overinvestment

For Hypothesis H1, the relative compensation of executives is used to replace the explanatory variables. Table 9 shows the robustness test results of Hypothesis H1.

**TABLE 9:** Regression results of overconfidence and overinvestment.

Variables	Coefficient	*T*-value	VIF
***OC*1**	0.0075***	4.3333	1.1213
***Top* 1**	–0.0044	–0.7113	1.3912
***Growth***	0.0070***	10.077	1.3811
***Size***	–0.0004	–0.5299	1.216
***Age***	−0.0009**	–4.954	1.4491
***Roe***	0.0362**	5.1657	1.1367
***Market***	–0.0013	–0.6909	1.4467
***Industry***		Control	
***Year***		Control	
***Constant term***	0.0523**	2.4232	
***F-value***		10.01	
***Sig.***		0.0000***	
***Durbin-Watson***		1.4652	
***Number of samples***		6,012	
***Adj.R* ^2^**		0.212	

***p < 0.01, **p < 0.05.

It can be seen from the results in Table 9 that the *Adj.R*^2^ is 0.212, indicating that all variables in H1 explain 21.20% of the overinvestment, and the model has a good goodness of fit. The *F-value* is 10.01 and the *Sig.* is 0.0000, which is significant at the 1% confidence level. All variables VIF did not exceed 2, indicating that there was no multicollinearity among the variables. The *Durbin-Watson* is 1.4652, indicating that there is no autocorrelation in the random error term. After replacing the measurement method of explanatory variables, the regression coefficient of managerial overconfidence (*OC*1) is significantly positive, and it is still significant at the 1% level, which is consistent with the previous regression results.

(2) Robustness test of the moderating effect of media reports on overconfidence and overinvestment

For hypotheses H2a and H2b, media reports were further introduced as moderating variables, and the interaction terms of positive and negative media reports and overconfidence were added into the models for regression, respectively. Table 10 shows the robustness test results of hypotheses H2a and H2b.

**TABLE 10:** Regression results of the moderating effect of positive and negative media reports.

Variables	Coefficient	*T*-value	VIF	Coefficient	*T*-value	VIF
***OC*1**	0.0075***	3.8434	1.0213	0.0076***	3.898	1.0362
***P*_*Media*_2**	−0.0142***	–4.4099	1.4254			
***P*_*Media*_2 × *OC*1**	0.0281***	5.7618	1.0618			
***N*_*Media*_2**				0.0024	0.8548	1.0236
***N*_*Media*_2 × *OC*1**				−0.0097**	–2.0579	1.432
***Top* 1**	–0.0008	–0.1139	1.0912	–0.0038	–0.5507	1.5212
***Growth***	0.0078***	8.9734	1.3611	0.0079***	9.0714	1.0611
***Size***	–0.0006	–0.6215	1.21	0.0011	1.1042	1.01
***Age***	−0.0007***	–3.6449	1.0491	−0.0008***	–4.1792	1.0241
***Roe***	0.0363***	4.2243	1.1387	0.0357***	4.3671	1.2987
***Market***	0.003	1.4512	1.2467	0.0011	0.5217	1.0234
***Industry***		Control			Control	
***Year***		Control			Control	
***Constant term***	0.0446*	1.6549	1.1469	0.0197	0.734	1.4345
***F-value***		0.0000***			0.0000***	
***Sig.***		8.11			7.76	
***Durbin-Watson***		1.4654			1.3462	
***Number of samples***		6,012			6,012	
***Adj.R* ^2^**		0.198			0.243	

***p < 0.01, **p < 0.05, *p < 0.1.

As can be seen from Table 10, for positive media reports, the *Adj.R*^2^ is 0.198, indicating that the degree of overexplaining of all variables in Hypothesis 2 is 19.80%, and the goodness of fit of the model is good. The *F-value* is 8.11 and the *Sig.* is 0.0000, which is significant at the 1% confidence level. The VIF of all variables did not exceed 2, indicating that there was no multicollinearity among the variables. The *Durbin-Watson* is 1.4654, indicating that there is no autocorrelation in the random error term.

The *Adj.R*^2^ of the regression of negative media reports is 0.243, indicating that the degree of explanation of all variables in Hypothesis 2 is 24.30%, and the goodness of fit of the model is good. The *F-value* is 7.76 and the *Sig.* is 0.0000, which is significant at the 1% confidence level. The VIF of all variables did not exceed 2, indicating that there was no multicollinearity among the variables. The *Durbin-Watson* is 1.3462, indicating that there is no autocorrelation in the random error term.

After substituting the measures of overconfidence and media reports, positive reports multipliers (*P*_*Media*_2 × *OC*1) and *Overinv* are significantly positively correlated at the 1% level. Negative media reports (*N*_*Media*_2 × *OC*1) and *Overinv* are significantly negatively correlated at the 5% level. The overall results are consistent with the previous results, indicating that the results are not random, and the assumptions are robust.

(3) Robustness test of the moderating effect of positive media reports under different marketization degrees

First, the robustness test of H3a is carried out, and the positive media reports are regressed. The results are shown in Table 11.

**TABLE 11:** Regression results of positive media reports under different marketizations.

Variables	Coefficient	*T*-value	VIF	Coefficient	*T*-value	VIF
***OC*1**	0.0107***	3.5544	1.1456	0.0066***	2.5913	1.6533
***P*_*Media*_2**	0.0011*	–0.2503	1.3216	−0.0294***	–6.3312	1.4123
***P*_*Media*_2 × *OC*1**	0.0044*	0.6039	1.0361	0.0523***	7.6994	1.3126
***Top* 1**	0.0015	0.136	1.2154	–0.0002	–0.022	1.4212
***Growth***	0.0106***	7.7045	1.3178	0.0064***	5.5587	1.3178
***Size***	0.002	1.2694	1.1179	–0.0019	–1.4315	1.5123
***Age***	−0.0007**	–2.1396	1.4123	−0.0008***	–3.0863	1.4231
***Roe***	0.0479***	3.6082	1.3127	0.0307***	2.6623	1.1367
***Industry***		Control			Control	
***Year***		Control			Control	
***Constant term***	–0.0193	–0.5152	1.5467	0.0909	1.1733	1.3256
***F-value***		27.34			19.24	
***Sig.***		0.0000***			0.0000***	
***Durbin-Watson***		1.3531			1.5628	
***Number of samples***		2,534			3,478	
***Adj.R* ^2^**		0.214			0.198	

***p < 0.01, **p < 0.05, *p < 0.1.

It can be seen from Table 11 that the *Adj.R*^2^ after regression of the low marketization level group and the high marketization level group are 0.214 and 0.198, respectively, indicating that the goodness of fit of the regression model is acceptable. The *F-value* were 27.34 and 19.24, respectively, and the *Sig.* were both 0.0000, which were significant at the 1% confidence level. The VIF of all variables does not exceed 2, and the *Durbin-Watson* are random error terms without autocorrelation. In high marketization regions, the regression coefficient between positive media reports and overconfidence (*P*_*Media*_2 × *OC*1) and overinvestment is much larger than that in low marketization regions, and it is significantly positive, which is consistent with the previous regression results.

Robustness test is carried out on the moderating effect of negative media reports under different marketization degrees, and the regression results are shown in Table 12.

**TABLE 12:** Regression results of negative media reports under different marketizations.

	Low marketization			High marketization		
Variables	Coefficient	*T*-value	VIF	Coefficient	*T*-value	VIF
***OC*1**	0.0112***	3.7125	1.5213	0.0062***	2.4199	1.5362
***N*_*Media*_2**	0.0130***	2.8906	1.4254	–0.0047	–1.2332	1.4254
***N*_*Media*_2 × *OC*1**	−0.0294***	–4.211	1.0295	0.005	0.7585	1.0295
***Top* 1**	–0.0012	–0.1074	1.2912	–0.0029	–0.3148	1.5712
***Growth***	0.0106***	7.7119	1.3671	0.0064***	5.6402	1.0631
***Sise***	−0.0039**	2.4375	1.217	–0.0004	–0.2688	1.0106
***Age***	−0.0007**	–2.22	1.4491	−0.0009***	–3.7048	1.0341
***Roe***	0.0489***	3.7203	1.1397	0.0316***	2.7258	1.4987
***Industry***		Control			Control	
***Year***		Control			Control	
***Constant term***	–0.0438	–1.186	1.1569	0.0625	0.8018	1.0345
***F–value***		16.75			15.28	
***Sig.***		0.0000***			0.0000***	
***Durbin-Watson***		1.4563			1.8755	
***Number of samples***		2,534			3,478	
***Adj.R* ^2^**		0.141			0.225	

***p < 0.01, **p < 0.05.

It can be concluded from Table 12 that the adjusted R2 after regression of the low marketization level group and the high marketization level group are 0.141 and 0.225, respectively, indicating that the goodness of fit of the regression model is acceptable. The VIF of all variables does not exceed 2, and the *Durbin-Watson* are small, indicating that there is no autocorrelation in the random error term. Under the low marketization level, the regression coefficient of negative media report interaction term (*N*_*Media*_2 × *OC*1) and overinvestment is significantly negative, which is consistent with the above regression results.

## Discussion

### Policy recommendations at the enterprise level

#### Strengthening managers’ self-learning and improvement

Studies have found that managers will have self-perception biases due to factors such as age, gender, and background, overestimating their own abilities and underestimating the probability of risk and failure. This kind of mentality will cause huge losses to the enterprise. In view of this, managers should improve their self-awareness, keep a clear head in business operations and treat them rationally, and avoid making irrational decisions such as overconfidence and overinvestment. Managers’ learning of industry professional theory and relevant knowledge of risk assessment should be strengthened. The ability of managers to self-reflect and summarize should be strengthened, to obtain lessons from failure and successful experience, and to maintain a clear understanding of themselves at all times.

#### Establishing a sound and scientific investment evaluation system

First of all, before making investment decisions, enterprises should scientifically and rationally analyze the prospects and rates of return of investment projects, so as to avoid managers making wrong investment decisions due to high investment enthusiasm and irrational psychology. Secondly, enterprises should strengthen the supervision of management, and constantly improve the mechanism of checks and balances of power, so as to avoid excessive power of managers. Finally, enterprises should continuously improve and perfect the promotion incentive mechanism and career development path for managers, and reduce excessive investment due to the utilitarian psychology of pursuing performance.

#### Paying attention to and treating media reports rationally

Enterprises should pay attention to and treat media reports correctly and rationally, and maintain a good and healthy relationship between the media, enterprises and the public. For negative media reports, enterprises should reflect on their own behavior in a timely manner, and strive to make up for the losses caused to the enterprises, shareholders. Managers should analyze and evaluate positive media reports objectively and rationally, and avoid being overwhelmed by positive reports, resulting in high investment enthusiasm and irrational behaviors such as excessive investment.

### Policy recommendations at the government level

#### Strengthening the media’s role in supervising enterprises

As a supplement to the capital market supervision mechanism, the government should make full use of the media’s public opinion advantage and play its role in external governance. The government should attach importance to and strengthen the media’s negative reports and supervision of enterprises, and urge administrative supervision departments to strictly supervise relevant behaviors. It can be seen from the research that the media mechanism and the marketization process are the relationship of substitution. The media can better play the role of corporate governance in regions with a low degree of marketization. Therefore, especially in areas with a low degree of marketization, the media should pay more attention to and strengthen the supervision of enterprises, carry out negative reports and expose illegal activities, and play the role of corporate governance.

#### Guiding the healthy and orderly development of the media industry

First, the government should create a good environment for the media, ensure the freedom and independence of the media industry, and put an end to the phenomenon of “government-controlled media.” Secondly, the government should guide the media industry to develop toward a healthier, more orderly, and more transparent development, reduce the phenomenon of media and enterprises colluding and mislead public opinion, and increase the punishment for media violations. In addition, with the rapid development of emerging media, the government should encourage traditional media to carry out industrialization reforms and pursue innovation and transformation in the context of big data.

### Policy recommendations at the media level

#### Continuously improving the industry self-regulation and supervision system

The media should always ensure its own objectivity, report and disclose corporate information from a neutral standpoint, and treat any events and news without bias or exaggeration. The media should present facts and evidence to the public, ensure the reliability and timeliness of reports, correct deviations in media reports from the source, and truly play the role of media and information bridges. The media system must attach importance to the supervision and management of the industry, improve the ability of self-supervision and self-discipline, maintain the advanced nature and purity of the media industry system, and improve the overall image and credibility of the media in the minds of the public.

#### Accelerating the innovative transformation of the industry

Under the continuous advancement of the era of big data, the emergence of many emerging media such as self-media has caused a huge impact on traditional media. The media should accelerate their own industrial transformation, actively innovate, and use the Internet to promote more comprehensive, faster, and more efficient dissemination of media reports, and further expand their coverage, so that news media can truly become civilians.

## Conclusion

This paper further explores the relationship between managers’ overconfidence, media reports and enterprise overinvestment, puts forward the hypothesis of this paper, and collects and organizes the relevant data of A-share listed companies from 2013 to 2021. Through empirical analysis, the influence of overconfidence on overinvestment and the moderating effect of positive and negative media reports on the relationship between the two are deeply analyzed, and the robustness test is carried out. Finally the following conclusions are drawn:

(1) There is a positive correlation between managers’ overconfidence and overinvestment. The higher the level of managerial overconfidence, the more likely it will lead the company to overinvest. Overconfident managers have a stronger sense of superiority, have strong egos and are overly optimistic about investment projects and business prospects, have high enthusiasm for investment, and underestimate or even ignore market risks. Therefore, overconfident managers will lead companies to invest in some non-quality projects, resulting in excessive investment, weakening enterprise value, and damaging shareholders’ interests.

(2) Positive media reports can positively moderate overinvestment caused by overconfidence, while negative media reports can alleviate and negatively moderate overinvestment caused by overconfidence. Positive media reports will cause managers to become more enthusiastic about investment, which is more likely to lead companies to overinvest. Negative media reports can seriously affect the reputation of companies and managers. In order to restore the enterprise image and reputation, managers will reduce their enthusiasm for foreign investment, and will be more prudent and conservative in their investment decisions. They will fully consider market risks, thereby reducing excessive investment behavior, using the correct investment direction and high investment efficiency to restore enterprise image and re-attract investors.

(3) Compared with areas with a low degree of marketization, positive media reports in areas with a high degree of marketization will more obviously aggravate the overinvestment caused by managers’ overconfidence. In regions with a low degree of marketization, negative media reports can better restrain the overinvestment caused by managers’ overconfidence. This shows that media governance and the process of marketization are substitutes. In regions with a low level of marketization, negative media reports can play a greater role, and can better negatively regulate excessive investment caused by managers’ overconfidence.

### Research limitations and future development

(1) At present, there is no standard and authoritative measure to measure “manager’s overconfidence.” This paper draws on other scholars to choose “personal background characteristics” as a substitute variable to measure the psychological degree of managers’ overconfidence, which has certain defects and is absolute.

(2) In this study, the selection of “media reports” only considers the paper media. With the advancement of science and technology in recent years, emerging media such as mass Internet have risen rapidly, and emerging media reports such as radio, TV, and online platforms such as TikTok or Weibo have also accounted for a large share. Not including emerging media is a shortcoming of this paper.

Based on the above deficiencies, prospects for more in-depth research in the future are put forward: evidence from other countries (United States, Europe) will be added to complement existing methods. Exploring the rationality of the method used in this paper and exploring a more optimized way are the future research priorities and trends in this field. In addition, in addition to traditional media, media report data from other channels such as the Internet and TV should also be considered. Therefore, in the era of big data and the emerging trend of emerging media, we will explore how countries around the world can more comprehensively include media report data and information, and strive to obtain more comprehensive and complete media report data.

## Data availability statement

The raw data supporting the conclusions of this article will be made available by the authors, without undue reservation.

## Author contributions

The author confirms being the sole contributor to this work and has approved it for publication.
